# The Efficacy of Percutaneous Patent Foramen Ovale Closure on Migraine: a Meta-Analysis of Randomized Controlled Trials and Observational Studies

**DOI:** 10.1155/2021/6643266

**Published:** 2021-03-04

**Authors:** Quan-Quan Zhang, Jia-Jie Lu, Man-Yun Yan, Xiao-Wei Hu, Yi-Ren Qin, Da-Peng Wang, Jian-Hua Jiang, Qi Fang, Hong-Ru Zhao

**Affiliations:** Department of Neurology, The First Affiliated Hospital of Soochow University, Suzhou 215006, China

## Abstract

**Objectives:**

Whether patent foramen ovale (PFO) closure is effective on migraine is controversial. This article was aimed at assessing the efficacy of PFO closure on migraine based on randomized controlled trials (RCTs) and observational studies.

**Methods:**

We searched PubMed, Embase, and Cochrane databases up to October 2020 evaluating PFO closure versus control in patients with migraine, then conducted a meta-analysis of all RCTs and observational studies, respectively. The main outcomes were (1) respond rate: complete cessation of migraine; (2) reduction in the frequency of migraine attacks per month; and (3) reduction in migraine days per month.

**Results:**

Seven studies (3 RCTs and 4 observational studies), containing 887 migraine patients, were identified. (1) The respond rate of PFO closure on migraine was significantly higher than control group both in RCT subgroup and observational studies subgroup (OR 3.86, 95% CI 1.35-11.04, *P* = 0.01 in RCTs; OR 8.28, 95% CI 2.31-29.67, *P* = 0.001 in observational studies). (2) Reduction in frequency of migraine attacks was higher in PFO closure group compared with control group in the RCT subgroup analysis (mean difference (MD) = 0.57, 95% CI 0.23-0.90, *P* = 0.0009). (3) Reduction in migraine days was also higher in PFO closure group compared with control group in the RCT subgroup analysis (MD = 1.33, 95% CI 0.35-2.31, *P* = 0.008).

**Conclusions:**

PFO closure might be suitable for migraine patients, especially for migraine with aura, by cessation of migraine headaches or reducing migraine attacks and migraine days.

## 1. Background

Migraine is a common recurrent and disabling primary headache, affecting almost 13% of the general population. In approximately 36% of patients, the migraine attack is preceded by an aura [1, 2]. Data for primary headache from Global Burden of Diseases, Injuries, and Risk Factors (GBD) 2016 lead to the conclusion that migraine is responsible for substantial burden of disease worldwide [3]. Multiple studies have reported a significant association between migraine, especially migraine with aura (MA) and patent foramen ovale (PFO) [4, 5], and the incidence of PFO in MA patients is about 50% [6]. The presence of right-to-left shunting (RLS) is revealed to be correlated with MA and its pathological hypothesis may include genetic influence and migraine attack triggered by vasoactive substances reaching the brain in a higher concentration [5]. Several studies have shown that the frequency of migraine attack of MA could be reduced by 70-80% after PFO closure in patients with other indications, such as stroke [7]. Furthermore, some observational studies have shown that migraine headaches improved significantly after PFO closure in patients of migraine with PFO [8–10], but three major RCTs evaluating PFO closure for the treatment of migraine, MIST, PRIMA, and PREMIUM, failed to meet their primary efficacy endpoint [11–13]. All three trials showed numerical benefits of PFO closure and two proved an advantage with a statistically significant difference, albeit only in secondary endpoints [11, 12]. Hence, the benefit of PFO closure for migraine is controversial. We conducted a meta-analysis to assess the efficiency of PFO closure in migraine patients on the basis of RCTs and observational studies in order to guide clinical practice.

## 2. Methods

### 2.1. Study Search Strategy

We performed a computerized search of the Cochrane Library, PubMed, Embase, Wanfang Patent Database (WFPD), Weip Database, and China National Knowledge Infrastructure databases (CNKI) through October 2020, using the following terms: “migraine” AND “patent foramen ovale” OR “PFO” AND “closure.”

### 2.2. Study Selection Criteria

The inclusion criteria were as follows: (i) randomized controlled trials (RCTs) and observational studies; (ii) comparison of the efficacy of PFO closure and drug treatment or sham surgeon procedure; (iii) participants were migraines with PFO; and (iv) the primary efficacy endpoint contained complete cessation of migraine, which we defined as respond rate. The secondary efficacy endpoint included the reduction in monthly migraine attacks and migraine days. The main exclusion criteria were as follows: (i) studies with incomplete data or unclear outcome; (ii) republished studies.

### 2.3. Data Extraction

Two investigators independently appraised the identified articles according to the above-mentioned inclusion criteria and resolved differences of opinion by consensus resolution or consulting a third participant in cases of disagreement. If any of these data were not available in the publications, further information was sought by correspondence with the authors or the reference. The two researchers extracted the following data independently: (i) basic information, such as the first author and publication time of the included studies; (ii) baseline characteristics of subjects, including sample size of each group, age of patients, detection method of PFO, and so on; (iii) specific intervention measures, follow-up time, and endpoints; and (iv) the key elements evaluating the quality of literature.

### 2.4. Study Quality Assessment

The Cochrane risk of bias tool was used to test the quality of RCTs, which included random sequence, distribution hidden, blind method, incomplete data report, selective reporting data, and other bias. If the indicator of the above evaluation item was judged as “yes,” it indicated a low risk of bias. If the evaluation item was judged as “no,” it indicated a high risk of bias, and the unclear or unknown risk of bias was judged as “unclear.” Disagreements during the process were resolved by discussion or determined by a third investigator. The Newcastle-Ottawa scale (NOS) was used to evaluate the methodological quality of case-control and cohort studies, and high-quality studies were classified as NOS ≥ 7.

### 2.5. Quantitative and Statistical Analysis

The Review Manager 5.3 Tests provided by the Cochrane website were used for statistical analysis. Categorical variables were presented as odds ratio (OR) and 95% confidence interval (CI), while continuous variables were presented as mean difference and 95% CI. Heterogeneity was assessed by Chi-squared test and *I*^2^ statistics. The random-effects models were used when *P* < 0.1 and *I* > 50%, suggesting a considerable heterogeneity in the included studies. The fixed-effect methods were used when *P* > 0.1 and *I*^2^ ≤ 50%. A two-sided *P* < 0.05 was considered significantly different.

## 3. Results

### 3.1. Search Results

After screening and assessing for eligibility, eleven studies were further investigated. Seven studies with a total of 887 patients were included finally, containing 3 RCTs [11–13] and 4 observational studies [10, 14–16]. The study selection process was described in the flow diagram (Figure 1).

### 3.2. Study Quality Assessment and Publication Bias

The bias risk assessment results of 3 RCTs are shown in Figure 2. All the RCTs were high-quality researches with low risk of bias. The NOS scores of 4 observational studies are listed in Tables 1 and 2. All observational studies were evaluated as high quality. 3 studies [10, 14, 15] scored eight points, and 1 study [16] scored seven. For all RCT outcome analyses, the heterogeneities were low or inexistence, as represented in Figures 2, 3 and 4, respectively, while, when we combined 4 observational studiess, the heterogeneity increased (*χ*^2^ = 6.87, *P* = 0.08, *I*^2^ = 56%, see Figure 5).

### 3.3. Patients and Study Characteristics

The characteristics of the included studies are described in Table 3. All participants had not been confirmed as symptomatic stroke or transient ischemic attack except that of Biasco et al. [14], which was not mentioned. Most of the studies included moderate to severe disabling, medication-refractory migraineurs, while in two studies [14, 15], it was not mentioned. A contrast transthoracic echocardiography (c-TTE)/transesophageal echocardiography (TEE) test [10, 12–16] or contrast transcranial Doppler (cTCD) measurements [10–12, 14–16] were performed to determine the presence of PFO and severity of an RLS.

### 3.4. Effect Analysis

#### 3.4.1. Respond Rate

The respond rate of PFO closure on migraine was analyzed in 7 studies (3 RCTs and 4 observational studies), with a total of 887 patients. The respond rate was evaluated as complete cessation of migraine at the end of follow-up. In the RCT subgroup, the estimated effect of PFO closure was reflected by a summary OR of 3.86 (95% CI, 1.35-11.04) using the fixed-effect model, in accordance with not evident statistical heterogeneity (*I*^2^ = 48%, *P* = 0.15). Moreover, the efficacy was significant (*P* = 0.01) (Figure 2). In the observational studies, the summary OR was 8.28 (95% CI, 2.31-29.67), with a relatively higher heterogeneity (*I*^2^ = 56%, *P* = 0.08); thus, we used a random-effect meta-analytical approach to combine the results of the individual studies. The efficacy was also significant (*P* = 0.001) (Figure 5).

#### 3.4.2. Reduction in Frequency of Migraine Attacks per Month

This study outcome was accessed only in the 3 RCTs. The reduction in monthly migraine attacks was significantly higher in PFO closure compared with the control group (MD = 0.57, 95% CI 0.23-0.90, *P* = 0.0009). And the trials were calculated as no statistical heterogeneity (*χ*^2^ = 0.38, *P* = 0.83, *I*^2^ = 0%) (Figure 3).

#### 3.4.3. Reduction in Migraine Days per Month

Reduction in monthly migraine days was also evaluated in RCTs but only in PRIMA and PREMIUM trials, while data from MIST trial was not available. There was a higher reduction of monthly migraine days in the PFO closure group compared with control group (MD = 1.33, 95% CI 0.35-2.31, *P* = 0.008). The statistical heterogeneity of the two trials was detected as inexistence (*χ*^2^ = 0.04, *P* = 0.85, *I*^2^ = 0%).

## 4. Discussion

Migraine is one of the most common neurological diseases, affecting around 13% of the general population [17], and was also one of the five leading causes of years of life lived with disability (YLDs) in 2016 [18], which brings a significant burden to society. Despite various prevention methods, medication only works for 30-50% of migraine sufferers [19]. Some studies had shown that there was a close relationship between migraine and PFO, especially MA [20, 21]. Further studies also suggested a positive impact for PFO closure on patients with migraine, suggesting a possible causal link between migraines and RLS via PFO [4, 22]. Three RCTs were conducted to evaluate the effect of PFO closure on migraine, all of which failed to meet their primary endpoints defined as migraine resolution or greater than 50% reduction in migraine days at one year [23]. However, two of the clinical trials showed significant benefits in secondary endpoints and in migraine subgroup patients [11, 12]. We conducted this study as a meta-analysis of randomized trials and observational studies to collect all available data on the yield of PFO closure in patients with migraine.

In the current studies evaluating the effect of PFO closure on patients with migraine, we totally analyzed 3 RCTs and 4 observational studies whose outcome assessments included complete migraine remission. The result showed the rate of disappearance of migraine was much higher after transcatheter closure compared with the control group, either in RCTs' or observational studies' subgroup analysis. Mainly based on 3 RCTs, we evaluated the outcomes of reduction in monthly migraine attacks and migraine days. The results also indicated that the reduction in monthly migraine attacks was higher in the PFO closure group compared with the control group. Similarly, reduction in monthly migraine days was also significantly better in the PFO closure group.

The respond rate describing as complete cessation of migraine headache in our meta-analysis was positive. This finding stood in contrast to results of the MIST trial [13], of which the primary efficacy endpoint, cessation of migraine headache 91 to 180 days after the procedure, was not reached. This discrepancy could be explained as follows. First, the possible reasons might be unusually high procedural complication and residual shunt rates, presumably due to the type of device used [4, 19]. Residual shunt may still cause headache attacks. Eyal et al. found that 6 months after PFO closure, 26% patients had residual RLS. Absence of RLS was associated with improvement in migraine burden by >50% [24]. Second, it is noted that in the MIST trial, after exclusion of 2 patients who were responsible for 20% of all headache days in the closure group during the analysis period, there would be a significant reduction in migraine days between the two groups.

In the PREMIUM trial, complete migraine remission for one year occurred in 10 patients (8.5%) in the PFO closure group versus 1 patient (1%) in the control group (*P* = 0.01). In the PRIMA trial, 4 of 40 patients (10%) in the PFO closure group were free of migraine attacks during 10-12 months compared with none among 41 controls (*P* = 0.055). Then, when we combined those migraine free patients in the treatment group and control group to meta-analyze in the 3 RCTs, we got positive results. The MIST and PRIMA trials were targeted for MA patients. In addition, the PREMIUM trial mainly demonstrated complete cessation of migraine attacks for subjects with frequent aura (15.4% versus 2.5%). We were encouraged by the conclusion, but it should not be overstated because complete freedom of migraine attacks was achieved mainly in MA patients [11–13], which was consistent with the analysis of Shi et al., where they found a higher incidence of symptom improvement in patients with MA, compared with patients who do not experience aura [4]. It is hoped that future trials may focus on PFO closure in a more selected patient population of migraine with frequent aura. Moreover, closing a PFO for migraine conveys the collateral benefit of lifelong protection against paradoxical embolism causing stroke, myocardial infarction, or peripheral ischaemia [25]. Device PFO closure is so easily accomplished that it can be referred to as mechanical vaccination against such events [26].

In our analysis, we have also found a significant improvement in the reduction in migraine attacks and migraine days per month associated with PFO closure. Elbadawi et al. conducted a meta-analysis of the 3 RCTs and concluded that PFO closure might be beneficial in migraine patients by reducing migraine attacks and migraine days, especially in patients whose majority of migraine attacks were with aura [27]. Our analysis reached a consensus with their conclusion. Again, the respective nonsignificant primary endpoints of the PRIMA and PREMIUM trials met statistical significance in the sister trial where they figured as secondary endpoints [28]. Ignoring what were primary and secondary endpoints, both PRIMA and PREMIUM proved a significant advantage [29]. Just as the United States Headache Consortium has recommended, the goals for efficacious migraine prevention were including a decrease in migraine attacks frequency by 50% as well as a decrease in intensity and duration [30, 31]. From this point of view, the 2 RCT trials have achieved the desired effect.

Although it is controversial that antiplatelet therapy for 3-6 months after device closure for the prevention of device-adherent thrombi may have potential therapeutic effect in reduction of migraine symptoms in some patients with PFO [21], Tarantini et al. conducted a mean follow-up of 51 months of percutaneous PFO closure on migraine for the treatment of structural cardiac disease, and the results showed the positive effect of PFO closure on migraine persisted at long-term follow-up, even after drug discontinuation [32]. Since most of the case series were unblinded and the duration of follow-up is relatively short, there is debate that placebo effect may be considered an explanation for the reported positive response [33]. Although this placebo response in the PREMIUM study is 32%, it is within the range of control arm responses observed in other studies of migraine-preventive therapy [11]. Schwerzmann et al. found that headache attacks in patients with migraine were reduced by >50%, whereas no reduction was observed in patients with nonmigraine headaches, which render a sole placebo effect unlikely [21]. By the same token, Elbadawi et al. conducted a sensitivity analysis including only sham-controlled studies in the 3 RCTs' meta-analysis, and results also showed improvement of primary outcome with PFO closure [27], which support that the effect is unlikely to be caused just by a placebo effect. Similarly, it should not be ignored that the control group may also have placebo effects on patients due to sham procedure.

Why patients with PFO have migraine or vice versa are mainly based on 2 possible theories? One theory is subclinical emboli, which could be mediated via RLS allowing microemboli to pass from the venous system to systemic circulation [10]. This microemboli is believed to trigger cortical spreading depression, which is considered a key effector in the pathogenesis of MA. Another possible mechanism is intermittent RLS caused by PFO, which allows some chemicals to circumvent the clearance metabolism of the lungs and directly enter the systemic circulation in high concentrations, then trigger cortical diffusion inhibition or irritate the trigeminal nerve and trigger a migraine [23, 34].

## 5. Limitations

Our study had several limitations. First, some of the included studies were retrospective, and memory bias was unavoidable. Second, the different devices employed in surgical procedures and the different protocols for assessing the outcomes may imply a higher heterogeneity among trials. Third, some endpoints were only applicable for evaluation in only a portion of the included studies, which would have restricted our analysis. Fourth, the participants in the included studies were recruited and enrolled prior to the availability of the latest better medications, such as calcitonin gene-related peptide (CGRP) or its receptor.

## 6. Conclusion

Some reviews of observational studies and RCTs in patients with migraine and PFO concluded that transcatheter PFO closure did not significantly reduce the frequency of migraine compared with conventional therapies and doubted that PFO closure was associated with an increased risk of incident adverse events. We reviewed dozens of retrospective observational studies of PFO closure for migraine that suggested a possible beneficial effect of PFO closure on migraine, especially for MA. There is a higher level of evidence support an association between the presence of a PFO and MA than the evidence of a causal link for PFO and migraine without aura. From the analysis of our study, we have reasons to be optimistic that a future randomized trial of PFO closure to reduce migraine should be conducted to identify the correct patient subset and evaluate the effect.

## Figures and Tables

**Figure 1:** Process of study selection. In total, 7 reports were included in the meta-analysis.

**Figure 2:** The forest plot describing respond rate of migraine patients in the PFO closure group compared with the control group in RCT subgroup analysis. Risk of bias describing the quality assessment of the 3 RCTs.

**Figure 3:** The forest plot describing the number of migraine attacks per month at the end of follow-up in the PFO closure group compared with the control group in RCT subgroup analysis.

**Figure 4:** The forest plot describing the number of migraine days per month at the end of follow-up in the PFO closure group compared with the control group in the 2 RCTs' meta-analysis.

**Figure 5:** The forest plot describing respond rate of migraine patients in the PFO closure group compared with the control group in observational studies subgroup analysis. The heterogeneity of the 4 observational studies was described as *P* = 0.08, *I*^2^ = 56%.

**Table 1:** NOS score of included case-control studies.

Score category	Score	Anzola	Vigna
Selection			
Is the case definition adequate	1	1	1
Representativeness of the cases	1	1	1
Selection of controls	1	1	1
Definition of controls	1	1	1
Comparability			
Comparability of cases and controls on the basis of the design or analysis	2	1	1
Exposure			
Ascertainment of exposure	1	1	1
Same method of ascertainment for cases and controls	1	1	0
Nonresponse rate	1	1	1
Total score		8	7

**Table 2:** NOS score of included cohort studies.

Score category	Score	Biasco	Rigatelli
Selection			
Representativeness of the exposed cohort	1	1	1
Selection of the nonexposed cohort	1	1	1
Ascertainment of exposure	1	1	1
Demonstration that outcome of interest was not present at start of study	1	1	1
Comparability			
Comparability of cohorts on the basis of the design or analysis	2	1	1
Outcome			
Assessment of outcome	1	1	1
Was followed up long enough for outcomes to occur	1	1	1
Adequacy of follow-up of cohorts	1	1	1
Total score		8	8

Note: A study can be awarded a maximum of one star for each numbered item within the Selection and Exposure categories/Selection and Outcome categories. A maximum of two stars can be given for Comparability.

**Table 3:** Baseline characteristics of 7 included studies.

Study	Year	*N*	Mean age	Inclusion patient	Control arm	Follow-up	Outcome assessment	Antiplatelet therapy after device closure
Anzola	2006	27/27	40/36	Migraine and PFO (stroke asymptomatic)	Medical therapy	12 m	Migraine free (migraine severity score equal to 0 at the end of follow-up), basal-end score	Aspirin 300 mg qd∗6 m
Biasco	2014	89/128	46.4/47.1	Migraine and PFO	Medical therapy	6 m, 12 m, yearly	Migraine resolution (subjective evaluation), MIDAS score, residual RLS	Aspirin 100 mg qd∗6 m Clopidogrel 75 mg qd∗3 m
Rigatelli	2010	40/46	38.9/40	Migraine (severe, disabling, medication-refractory migraine) and PFO (stroke asymptomatic)	Medical therapy	12 m	Migraine reduction(0%, 25%, 50%, 100%), MIDAS reduction	None
Vigna	2009	53/29	42/43	Migraine (moderate to severe) and PFO (subclinical brain MRI lesions)	Medical therapy	6 m	Disappearance and >50% reduction of total and disabling attacks, aura reduction	Aspirin 100 mg qd∗6 m Clopidogrel 75 mg qd∗3 m
MIST	2007	74/73	44.3/44.6	MA (failed ≥ 2 classes of prophylactic treatments) and PFO (moderate or large RLS)	Sham procedure	3 m, 6 m	Primary efficacy end point: migraine headache cessation; Secondary efficacy end points: change in the frequency of migraine attacks, HIT-6 score, MIDAS	Aspirin 75 mg qd∗3 m Clopidogrel 75 mg qd∗3 m
PRIMA	2016	53/54	44/43	MA (unresponsive to preventive medications) and PFO	Medical management	12 m	Primary endpoint: change in migraine with and without aura days; Secondary endpoints: change in migraine attacks with aura or without aura, and change of days with acute migraine medication use Others: MIDAS, SF12 Mental Component score	Aspirin 75 − 100 mg qd∗6 m Clopidogrel 75 mg qd∗3 m
PREMIUM	2017	123/107	43/44	Migraine (failed at least 3 migraine-preventive medications) and PFO (significant RLS)	Medical therapy with a sham procedure	12 m	Primary endpoint: the responder rate for a 50% reduction in migraine attacks (with or without aura) Secondary endpoints: decrease of migraine days per month	None, only Preventive therapy

Headache Impact Test-6, HIT-6; Migraine with Aura, MA; Migraine Disability Assessment Survey score, MIDAS; Patent Foramen Ovale, PFO; Right-to-Left Shunting, RLS.

## Data Availability

All studies and data can be obtained from the Cochrane Library, PubMed, Embase, Wanfang Patent Database (WFPD), Weip Database, and China National Knowledge Infrastructure databases (CNKI).
